# The Effect of Soluble RAGE on Inhibition of Angiotensin II-Mediated Atherosclerosis in Apolipoprotein E Deficient Mice

This article has been retracted.

**DOI:** 10.1371/journal.pone.0069669

**Published:** 2013-08-01

**Authors:** Dajeong Lee, Kyung Hye Lee, Hyelim Park, Soo Hyuk Kim, Taewon Jin, Soyoung Cho, Ji Hyung Chung, Soyeon Lim, Sungha Park

**Affiliations:** 1 Graduate Program in Science for Aging and Yonsei Research Institute of Aging Science, Yonsei University, Seoul, Republic of Korea; 2 Medical Science Research Institute, Kyung Hee University Medical Center, Seoul, Republic of Korea; 3 Cardiovascular Research Institute, Yonsei University College of Medicine, Seoul, Republic of Korea; 4 Division of Cardiology, Yonsei University College of Medicine, Seoul, Republic of Korea; 5 Severance Integrative Research Institute for Cerebral and Cardiovascular Diseases, Yonsei University College of Medicine, Seoul, Republic of Korea; 6 Brain Korea 21 Project for Medical Science, Yonsei University, Seoul, Republic of Korea; Harvard Medical School, United States of America

## Abstract

**Background:**

The cross talk between RAGE and angiotensin II (AngII) activation may be important in the development of atherosclerosis. Soluble RAGE (sRAGE), a truncated soluble form of the receptor, acts as a decoy and prevents the inflammatory response mediated by RAGE activation. In this study, we sought to determine the effect of sRAGE in inhibiting AngII-induced atherosclerosis in apolipoprotein E knockout mice (Apo E KO).

**Methods and Results:**

9 week old Apo E KO mice were infused subcutaneously with AngII (1 µg/min/kg) and saline for 4 weeks using osmotic mini-pumps. The mice were divided into 4 groups 1. saline infusion and saline injection; 2. saline infusion and sRAGE injection; 3. AngII infusion and saline injection; 4. AngII infusion and sRAGE injection. Saline or 0.5 µg, 1 µg, to 2 µg/day/mouse of sRAGE were injected intraperitoneally daily for 28 days. We showed that atherosclerotic plaque areas in the AngII-infused Apo E KO mice and markers of inflammation such as RAGE, ICAM-1, VCAM-1, and MCP-1 were increased in aorta compared to that of the Apo E KO mice. However, the treatment of 0.5 µg, 1 µg, and 2 µg of sRAGE in AngII group resulted in the dose-dependent decrease in atherosclerotic plaque area. We also demonstrated that sRAGE decreased RAGE expression level as well as inflammatory cytokines and cell adhesion molecules in AngII or HMGB1 treated-rat aorta vascular smooth muscle cells.

**Conclusion:**

The results demonstrated that partical blockade of RAGE activation by sRAGE prevent AngII -induced atherosclerosis. Therefore these results suggested that first, RAGE activation may be important in mediating AngII-induced atherogenesis, and second, AngII activation is a major pathway in the development of atherosclerosis. Taken together, results from this study may provide the basis for future anti- atherosclerotic drug development mediated through RAGE activation.

## Introduction

Activation of the renin-angiotensin system (RAS)-signaling pathway, through the activation of the NADPH oxidase system, results in increased oxidative stress and vascular inflammation and has a significant role in the pathogenesis of atherosclerosis. Previous studies have shown that activation of RAS signaling is associated with increased expression of the Receptor for Advanced Glycation Endproducts (RAGE) at the site of vascular inflammation [1], [2].

RAGE is an important endogenous pattern recognition receptor important for initiation of innate immune responses, and is a member of the immunoglobulin superfamily of cell surface molecules specific for diverse endogenous ligands [3], [4]. Activation of RAGE by ligands such as HMGB1, S100A/calgranulin, and advanced glycation end products is associated with induction of oxidative stress, increased inflammatory cytokines, and recruitment of proinflmmatory cells [5], [6]. RAGE signaling has been linked to various chronic inflammatory diseases such as diabetes, atherosclerosis, and inflammatory renal disease [7], [8]. Thus, the increase in damaged self-proteins during the initiation of vascular inflammation and atherogenesis may result in RAGE activation-mediated inflammation. Angiotensin II (AngII), through activation of NADPH oxidase, increases oxidative stress and vascular inflammation and is known to accelerate the development of atherosclerosis [9], [10]. However, there have been no reports regarding the role of RAGE during the progression of AngII-mediated atherosclerosis. Prior studies have shown that infusion of angiotensin II for 4 weeks in Apo E knockout mice is associated with acceleration of atherosclerosis beyond that observed in untreated Apo E knockout mice [11].

Therefore, in this study, we sought to determine the inhibitory effect of soluble RAGE (sRAGE), a decoy receptor that blocks RAGE activation and inhibits inflammatory responses mediated by RAGE activation, in an AngII-induced atherosclerosis model using Apolipoprotein E knockout (Apo E KO) mice.

## Materials and Methods

### Expression and Purification of sRAGE-Fc Fusion Protein

The purified mouse sRAGE-Fc fusion protein was purchased from A&R Therapeutics (Daejeon, Republic of Korea) for the experiment. Briefly, For the sRAGE-Fc construction, a leader sequence (gene ID: K02149; protein: AAA51633); mouse IgG H chain (primer set: 5′-ATAGGCTAGCGCCACCATGGGATGG-3′, 5′-TGTGTGAGTTTTGTCCGAGTGGACA TCTGT-3′), a.a 23–341 of mouse sRAGE (primer set: 5′-GGTCAGAACATCA CAGCCCGG ATTG-3′, 5′-TGTGTGAGTTTTGTCCCCCATGGTGCAAGA-3′), and the human IgG1 Fc region (primer set: 5′-GGCTAGCGTACCCAGCCCAGACTC-3′, 5′-CCAGCTCGAGCTATTTACCCGGAGACAG-3′) were amplified, and the overlap extension PCR was performed. To express the desired domain, PCR product was treated with SfiI and ligated into pYK 602-His vector (vector constructed by KRIBB). To express the mRAGE-Fc, Mouse sRAGE-Fc was transfected into HEK293E cells and collected supernatants every other day. To purify, a protein A-Sepharose column (Amersham Biosciences, Piscataway, NJ, USA) was used according to the manufacturer’s instructions. The purified recombinant sRAGE was dialyzed with PBS, analyzed by SDS-PAGE. After quantification, mRAGE was aliquoted and stored at −70°C for experiment. And analysis with the *Limulus* amebocyte lysate test kit (Cape Cod, East Falmouth, MA, USA) was performed to examine the endotoxin level.

### Animal Studies

Apo E KO male mice on a C57BL/6J background were obtained from the Jackson Laboratory (Bar Harbor, ME, USA) and all animal experiments conformed to the *Guide for the Care and Use of Laboratory Animals* that was published by the US National Institute of Health (NIH Publication No. 8523, revised 1985). 9-week-old Apo E KO mice were anaesthetized by intraperitoneally injection of zoletil (30 mg/kg) and xylazine (10 mg/kg), and then were infused subcutaneously with AngII (Sigma, St. Louis, USA) at a concentration of 1 µg/min/kg and saline for 4 weeks using osmotic mini-pumps (Alzet, model 2004; flow rate = 0.25 µl/hour). Mice were divided into 4 groups: 1. saline infusion and saline IP injection; 2. saline infusion and sRAGE IP injection (A&R Therapeutics, Daejeon, Republic of Korea); 3. AngII infusion and saline IP injection; 4. AngII infusion and sRAGE IP injection. sRAGE was injected daily for 28 days and the concentration of sRAGE varied from 0.5 µg, 1 µg, to 2 µg/day/mouse for each group to determine dose responsiveness (N = 10 for each groups).

After waiting for 28 days after the initial injection period, the animals were sacrificed for the necessary analysis. The animals were fed a standard diet *ad libitum*, had free access to water, and were housed in a room with 12 hours of light/dark cycle with a maintained temperature of 25°C for 9 weeks. All animal studies and post-mortem procedures were approved by the Institutional Animal Care and Use Committee of Yonsei University (Approval reference number: 2010-0310, 2011-0008).

### Determination of Blood Pressure

For the blood pressure determination, the mice that were used from for the blood pressure measurement were exposed to the same treatment protocol but were a separate group of mice from the animals sacrificed for pathologic assessment and immunohistochemical assessment. Briefly, 9-week-old Apo E KO mice were anaesthetized by intraperitoneally injection of zoletil (30 mg/kg) and xylazine (10 mg/kg), and then were infused subcutaneously with AngII (Sigma, St. Louis, USA) at a concentration of 1 µg/min/kg and saline for 4 weeks using osmotic mini-pumps (Alzet, model 2004; flow rate = 0.25 µl/hour). Mice were divided into 3 groups: 1. saline infusion and saline IP injection (N = 7); 2. AngII infusion and saline IP injection (N = 7); 3. AngII infusion and 2 µg/day of sRAGE IP injection for 28 days (N = 7). Systolic and diastolic blood pressure was measured in live mice by a non-invasive approach using a validated tail-cuff system that relies on volume pressure recording technology (BP-2000, Visitech Systems, Apex, NC, USA). Blood pressure was monitored on the 55^th^, 56^th^ day of the 8weeks experimental period. The chamber was kept at 35–36°C and the equipment was set for a maximum inflation pressure of 180 mmHg. Mice were placed in the restrainers several times before the measurements for acclimatization to the environment. All mice were first acclimated to the blood pressure measurements for 3 days (these data were discarded) and then the blood pressure was determined as the average measurement of the subsequent 2 days. For the blood pressure measurement protocol on each day, after the initial acclimatization of the mice for five cycles, the blood pressure was measured for 10 cycles and the average measurement was derived.

### Analysis of Atherosclerotic Lesion Area

Eight weeks after the AngII infusion, mice were anaesthetized by intraperitoneal injection of zoletil (30 mg/kg) and xylazine (10 mg/kg), and then hearts and aortas were perfused with phosphate-buffered saline (PBS) by cardiac puncture. Hearts were removed by cutting the ascending aorta and fixing in 4% (v/v) formalin for at least 24 hours. Aortas were dissected from the proximal ascending aorta and cut at the branch point. Adventitial fat was removed from aorta. Fixed aortas were opened longitudinally and stained with Oil Red-O solution for 12 hours, washed gently with distilled water, and photographed after pinning onto silicone plates. Formalin-fixed hearts were embedded in OCT compound (Leica biosystems, NUSSLOCH, Germany) and stored at −80°C. Frozen heart tissue was cut into 10 µm sections beginning with the lower portion of the heart until the aortic sinus was visible, then placed on tissue section polysine-coated slides (Thermo scientific, Hudson, NH, USA), and stained with Oil Red-O for 12 hours, washed with distilled water briefly, and photographed by microscopy. Lesional areas of whole aortas and plaques of aortic sinuses were calculated using the *Image J* program (National institutes of Health, USA; http://rsb.info.nih.gov/ij). Oil Red-O stained plaques were imaged from seven different animals, then data were averaged.

### Immunohistochemistry

Mouse aortas were removed from the heart and placed into PBS; adipose tissue was removed in situ. Segments of aortas were fixed in 10% (v/v) formalin solution and immersed in OCT compound, and stored at −80°C. Aorta cross sections (5 µm) were cut at the ascending aorta and the infrarenal abdominal aorta (2–3 mm below the renal artery) and incubated at 45°C for 12 hours to allow tissue to adhere to the slide. To stain with anti-RAGE, anti-MCP-1 (abcam®, Cambridge, UK), anti-ICAM-1, or anti-VCAM-1(Santa Cruz Biotechnology Inc., USA), sections were incubated with primary antibodies at 4°C for overnight, followed by fixation in acetone at −20°C for 10 minutes. Primary antibodies were used at1∶100. Stained slides were washed in PBS then incubated with biotinylated polyclonal secondary antibodies, and the slides were visualized using 3,3′-diaminobenzidine before glycerol gelatin mounting (Sigma, St. Louis, USA). Stained slides imaged from seven different animals were photographed by microscopy and were analyzed using the *Image J* program (National institutes of Health, USA; http://rsb.info.nih.gov/ij).

### RNA Extraction from Mouse Aorta Tissues and Reverse Transcription PCR

The expression levels of various genes were analyzed by reverse transcription-polymerase chain reaction (RT-PCR). Mouse aortas were removed from the heart and were stored in RNAlater Tissue Protect solution (QIAGEN, Mainz, Germany). Total RNA was isolated from aorta tissue using RNA isolation from the fibrous tissue kit (QIAGEN, Mainz, Germany). Complementary DNA (cDNA) was generated with the Reverse Transcription System (Bioneer, Seoul, Republic of Korea) according to the manufacturer’s instructions. 1 µg of total RNA was reverse-transcribed in a 20 µl reaction, with cDNA pre-mixed and 0.5 µg oligo-(dT) 15 primer at 42°C for 5 minutes. The reaction was terminated by heating at 90°C for 1 hour.

PCR was performed with the AccuPower PCR Premix (Bioneer, Seoul, Republic of Korea) and amplification conditions were as follows: reaction volume, 20 µL; primer, 10 pM; and template genomic DNA 1 µg. PCR was carried out in a thermal cycler using the following conditions: 95°C for 3 minutes, 95°C for 1 minute and then individual conditions for each gene. All PCR products were separated by electrophoresis on 1% agarose gels and visualized using staining with Gel-red (Biotium, Hayward, CA, USA) by Gel-Doc (Bio-Rad, Hercules, CA, USA).

The mouse gene primer sequences used for PCR were: mRAGE, forward 5′-CCTGGGTGCTGGTTCTTGCTCT-3′ and reverse 5′-GATCTGGGTGCTCTTACGGTCC-3′ (nucleotides 31–52 and 12091-230 in GenBank accession no. L33412); mICAM-1, forward 5′- GAGAGTGGACCCAACTGGAA-3′ and reverse 5′- CTTTGGGATGGTAGCTGGAA-3′; mVCAM-1, forward 5′- CCCAAGGATCCAGAGATTCA-3′ and reverse 5′- ACGTCAGAACAACCGAATCC-3′ [12]; mMCP-1, forward 5′- GGCTCA GCCAGATGCAGTTAA-3′ and reverse 5′- GTGAATGAGTAGCAGCAGGTGAGT-3′ (nucleotides 154–174 and 181–204 in GenBank Ref NM011333); and mGAPDH, forward 5′- AATGCATCCTGCACCACCAACTGC-3′ and reverse 5′- GGAGGCCATGTAGGCCATGAGGTC-3′ [13]. All samples were measured in triplicates for statistical analysis.

### Quantitative Real-Time PCR

PCRs were performed on LightCycler®480II System using the LightCycler® 480 SYBR green I master mix (Roche Diagnostics, Mannheim, Germany) according to the manufacturer’s instructions. The reaction mixtures conditions were as follows: final volume, 20 µL; cDNA, 500 ng;, 1 and forward and reverse primer, 10 pM. After pre-incubation at 95°C for 10 minutes, we performed 45 PCR cycles, each consisting of a denaturation step (95°C for 10 seconds) and an annealing step (58°C for 25 seconds). The intensity of the expression of each gene quantitated using LightCycler®480 Software 1.5.0 (Roche Diagnostics, Mannheim, Germany). Values were expr essed in arbitrary units. Relative values of mRNA levels were determined by that of GAPDH gene, and expressed as fold change over the control.

The mouse gene primer sequences used for PCR were: mRAGE, forward 5′-AAC ACA GCC CCC ATC CAA-3′, and reverse, 5′-GCT CAA CCA ACA GCT GAA TGC-3′ [14]; mICAM-1, forward 5′-CGC TGT GCT TTG AGA ACT GTG-3′ and reverse 5′-ATA CAC GGT GAT GGT AGC GGA-3′ [15]; mMCP-1, forward 5′-CTG AAG CCA GCT CTC TCT TCC T-3′ and reverse 5′-CAG GCC CAG AAG CAT GAC A-3′ [16] and mGAPDH, forward 5′-CAT GGC CTT CCG TGT TCC TA-3′and reverse 5′-GCG GCA CGT CAG ATC CA-3′ [17]. All samples were measured in triplicates for statistical analysis.

### Cell Culture and Treatment

Rat aorta vascular smooth muscle cells (VSMCs) were purchased from Biobud (Seongnam-si, Gyeonggi-do, Republic of Korea). Cells were cultured in Dulbecco’s Modified Eagle’s Medium (DMEM; Hyclone, Thermo Fisher scientific Inc., USA) containing 10% fetal bovine serum (FBS), Penicillin (10,000 Units/mL) and Streptomycin (10,000 µg/mL) in a humidified incubator at 37°C under an atmosphere of 5% CO_2_ and 95% air. All the experiments were performed with cells at the 6^th^ passage and incubated for 24 hours in serum-free medium before treatment. The cells were incubated with Ang II (100 nM) or sRAGE (0.5, 1, 2 µg/ml) for 24 hours and followed by HMGB1 (1 µg/ml) for 15 minutes before the end of the incubation period. Human recombinant HMGB1 was purchased from A&R Therapeutics (Daejeon, Republic of Korea).

### Western Blot Analysis

Mouse aortas were removed from the heart and homogenized immediately and lysed with RIPA buffer (Biosesang, Seongnam-si, Gyeonggi-do, Republic of Korea) containing a protease inhibitor cocktail (Calbiochem, Darmstadt, Germany). Cells were washed twice with cold PBS and lysed using the same buffer as aorta tissues. The protein concentration was measured by bicinchoninic acid protein assay. Equal amounts of total protein samples were loaded and separated by 10%–12.5% sodium dodecyl sulfate-polyacrylamide (SDS-PAGE) gel and electro-blotted to a polyvinylidene difluoride membrane. The membranes were blocked by Tris-buffered saline-Tween 20 (TBS-T, 0.1% Tween 20) containing 10% non-fat dried milk at room temperature for 1 hour and membranes were washed twice with TBS-T and anti-RAGE, anti-ICAM-1, anti-MCP-1, or anti-TNF-α(abcam®, Cambridge, UK); primary antibodies were incubated overnight at 4°C. Membranes were then washed with TBS-T and incubated with horseradish peroxidase-conjugated secondary antibody at room temperature for 1 hour. Signals were visualized using enhanced chemiluminescent detection (Millipore Corporation, Billerica, MA, U.S.A.). All samples were measured in triplicates for statistical analysis.

### Statistical Analysis

Data were expressed as the mean ± SD. ANOVA with Bonferroni’s correction were used to compare the means of two numeric values. Data analyses were done with commercially available GraphPad Prism 5 software. *p*-values*<*0.05 were considered statistically significant.

## Results

### Infusion of AngII Accelerates Atherosclerosis

To assess the activation of AngII with or without sRAGE, we generated an atherosclerosis model in Apo E KO mice over a period of 8 weeks. Mortality in the AngII-infused Apo E KO mice significantly higher compared to Apo E KO mice injected with saline (*p*-value = 0.013). However, there was no significant difference in mortality between Apo E KO mice injected with saline and AngII-infused Apo E KO mice that received sRAGE injection (*p*-value = 0.103). Although statistically non-significant, there was a tendency for the sRAGE injection group to have better survival compared to the angiotensin II infusion group (*p*-value = 0.220) (Figure 1A).

**Figure 1:** Survival and Development of Atherosclerotic Lesions in Apo E KO mice with AngII-induced atherosclerosis. A. Survival graph of Angiotensin II-induced atherosclerosis in Apo E KO mice with saline injection, AngII-infused, and AngII with sRAGE-treated groups. B. Immunohistochemistry sections of aorta (left =  ascending aorta, right =  infrarenal abdominal aorta) staining for inflammation markers (RAGE, ICAM-1, VCAM-1, and MCP-1) from Apo E KO mice saline injection and AngII-induced atherosclerotic Apo E KO mice (magnification: x10 and below RAGE data: x20). C. Decreased intensity in atherosclerotic areas of sRAGE-treated AngII-induced Apo E KO mice compared to AngII-induced Apo E KO mice (n = 7). The positive stain is expressed in arbitrary units normalized against a control. *p<0.01, Scale bar = 200 µm.

To check whether activation of NF-κB associated cell adhesion molecules and cytokines are associated with atherosclerosis formation with AngII treatment, cell adhesion molecules and cytokines were examined by immunohistochemistry in Apo E KO mice under several conditions at both the ascending aorta and the infrarenal abdominal aorta (Figure 1B). As activation of RAGE is known to increase inflammation markers and adhesion molecules [6], we chose representative cytokines and adhesion molecules for assessment. Aortic arches for experiments were collected and Cryo-sections were made for immunohistochemistry. Serial sections were stained and analyzed to detect the following markers of inflammation; RAGE, ICAM-1, VCAM-1, and MCP-1. Inflammatory markers were markedly increased in AngII-infused Apo E KO mice, whereas 2 µg of sRAGE injection was associated with significant reduction in the expression of inflammatory markers. Use of 0.5 µg or 1 µg of sRAGE also produced a concentration-dependent reduction in these inflammatory markers (Figure 1C).

### sRAGE Prevents AngII-induced Atherosclerotic Plaque Formation

As plaque formation is an important phenomenon in the atherosclerotic progress, we examined lesion progression in the aorta. Atherosclerotic lesion areas were markedly increased in AngII-infused mice compared to untreated controls, but sRAGE injection showed a marked reduction in atherosclerotic plaque areas, which were detected by Oil Red-O staining of en face and aortic sinuses (Figure 2 and 3). Oil Red-O staining of whole aortas showed more than a 2.5-fold increase in the atherosclerotic plaque area in AngII-infused Apo E KO mice compared to age-matched, untreated Apo E KO animals. In contrast, treatment with 2 µg of sRAGE resulted in a 70% decrease in the atherosclerotic plaque area as compared to mice that received only AngII-infusion (Figure 2). Quantitation of staining results is shown in Figure 2B. We injected lower doses of sRAGE, and found that injection of either 0.5 µg or 1 µg of sRAGE also resulted in a significant dose-dependent reduction in atherosclerotic plaque area to approximately 50%and 60%of that seen in mice that received AngII, respectively. Increased atherosclerosis was also distinct at the aortic sinus in the AngII-infused group, in which the lesion area was increased by over 12-fold compared to untreated Apo E KO mice. The administration of sRAGE decreased the average lesion area by 80% compared to the AngII-infused Apo E KO mice (Figure 3A and 3B). These findings suggest that sRAGE inhibits the development of AngII-mediated atherosclerosis.

**Figure 2:** Quantification of Atherosclerotic Lesions. A. Development of atherosclerotic plaque areas in en face aortas (n = 7, representative picture) stained with Oil Red-O stain from Apo E KO mice. B. The percent of atherosclerotic plaque area in the Apo E KO saline injection and in mice that received infusions of AngII with or without various doses of sRAGE. Relative quantification (% plaque area) was performed. *p<0.05 and **p<0.01.

**Figure 3:** Quantification of Atherosclerosis. A. Photomicrographs of atherosclerotic lesions from aortic sinuses of Apo E KO saline injection mice, AngII infused, and AngII infused with various doses of sRAGE (n = 7); scale bar, 200 µm. B. Quantitative data, *p<0.01.

### sRAGE Decreases Expression of Inflammation Markers and Adhesion Molecules

We next used whole aorta tissue lysates to measure the representative protein expression and mRNA levels of proteins as downstream targets of RAGE activation, such as the inflammatory marker MCP-1 and adhesion molecule ICAM-1 (Figure 4 and 5). Western blotting showed increased expression of RAGE, ICAM-1, and MCP-1 in AngII-infused Apo E KO mice. Treatment with sRAGE significantly decreased inflammatory markers in a concentration-dependent manner. In mice treated with 2 µg/ml of sRAGE, there was a significant reduction in the expression of RAGE, ICAM-1, and MCP-1 (Figure 4A and 4B). Similar findings were also observed when RT-PCR (Figure 5A) and quantitative Real-time PCR (Figure 5B) were performed for the expression of RAGE, ICAM-1, and MCP-1in AngII-infused Apo E KO mice with or without sRAGE. Protein and mRNA expression data demonstrate that increased levels of inflammatory markers induced by AngII can be significantly inhibited by RAGE blockade.

**Figure 4:** Effect of sRAGE in Apo E KO mice on Expression of Cytokines and Adhesion Molecules. A-B. Apo E KO mice infused with AngII were treated with various concentrations of sRAGE. Expressions of RAGE, ICAM-1 and MCP-1 were detected by western blot. The optical density is expressed in arbitrary units normalized against β-actin control. Data in histograms represent mean ± SD from individual 3 experiments. Lane 1, saline injection; lane 2, infusion of AngII; lane 3, infusion of AngII with 0.5 µg/day of sRAGE; lane 4, infusion of AngII with 1 µg/day of sRAGE; lane 5, infusion of AngII with 2 µg/day of sRAGE, *p<0.01.

**Figure 5:** Effects of sRAGE on mRNA Levels in Aorta of AngII-induced Apo E KO mice. A. Reverse transcription PCR analysis of RAGE, ICAM-1 and MCP-1 gene expression. Data in histograms represent mean ± SD from 3 experiments. Lane 1, saline injection; lane 2, infusion of AngII; lane 3, infusion of AngII with 0.5 µg/day of sRAGE; lane 4, infusion of AngII with 1 µg/day of sRAGE; lane 5, infusion of AngII with 2 µg/day of sRAGE. B. RAGE, ICAM-1 and MCP-1 mRNA expression level were determined by Real-Time PCR. Results are means ± SD from 3 experiments each performed in duplicate. *p<0.05, **p<0.01, *** *p*<0.001 and ns = non-significant.

### sRAGE Decreases Inflammation in Rat Aorta Vascular Smooth Muscle Cells

We first investigated whether sRAGE could inhibit expression of RAGE protein levels in VSMCs treated with AngII or HMGB1. Quantitative western blot analysis revealed that HMGB1 or AngII upregulated RAGE expression respectively compared to control VSMCs and HMGB1 with AngII showed a synergistic effect on RAGE expression. However, 0.5–2 µg/ml of sRAGE significantly decreased the AngII/HMGB1-induced RAGE expression by approximately 1.3-fold. We next investigated the effects of sRAGE on ICAM-1, MCP-1, and TNF-α protein levels. In agreement with our previous results, 0.5–2 µg/ml of sRAGE blocked AngII-induced activation of each of the above-mentioned markers by approximately 1.5-fold (Figure 6A and 6B).

**Figure 6:** Effect of sRAGE in Rat Aorta Vascular Smooth Muscle Cells. Western blot analysis showing expression of A, RAGE inflammation receptor protein, ICAM-1, MCP-1, and TNF-α; and B, Quantitative data from panel A. Expression of RAGE, ICAM-1, MCP-1, TNF-α, and β-actin were detected by western blot. Lane 1, control; lane 2, AngII-treated for 24 hours (100 nM); lane 3, HMGB1 treated for 15 minutes (1 µg/ml); lane 4, AngII plus HMGB1; lane 5, AngII plus HMGB1 and sRAGE (0.5 µg/ml); lane 6, AngII plus HMGB1 and sRAGE (1 µg/ml); lane 7, AngII plus HMGB1 and sRAGE (2 µg/ml); lane 8, treatment with sRAGE alone at 2 µg/ml. The optical density is expressed in arbitrary units normalized against a control. Data in histograms represent mean ± SD from 3 experiments. *p<0.01 vs control, ^†^ *p*<0.01 vs lane 4, ^#^ *p*<0.01 vs lane 4, ns = non-significant.

### Association AngII and Blood Pressure

The results from the mice tail blood pressure at the 55,56^th^ day of experiment showed that compared to Apo E knockout mice injected with saline (group 1), mice chronically infused with Ang II(group 2) were associated with significant increase in the systolic and diastolic blood pressure (*p<0.05). However, the systolic and diastolic blood pressure between group 2 and mice infused with AngII and injected with 2 µg/day of SRAGE (group 3) was not significant.

## Discussion

Activation of the renin-angiotensin-aldosterone (RAS) system is important in the pathogenesis of cardiovascular disease. Evidence from numerous basic and clinical studies has unequivocally demonstrated the clinical benefit of blocking RAS activation on improvement of the prognosis of cardiovascular disease [18], [19]. Angiotensin II, through the activation of the NADPH oxidase, may increase the degree of oxidative stress and vascular inflammation, which contributes to the pro-atherogenic effect of angiotensin II [20], [21]. Studies have shown that infusion of angiotensin II for 4 weeks in Apo E knockout mice is associated with acceleration of atherosclerosis beyond that of the control Apo E knockout mice [11]. Infusion of angiotensin II was also associated with neointimal proliferation of the vessel wall (Figure 1B) which was attenuated by sRAGE administration. There are several studies to support this result, in which NADPH oxidase inhibitor have been shown to suppress the angiotensin II induced neointimal formation [22], [23].

RAGE is a multi-ligand signal transduction receptor for AGEs, HMGB1, and S100/calgranulin. This receptor is an important mediator of innate immune responses to endogenous ligands, and is thus, known as an *alarmin* [5], [24]. RAGE activates inflammatory cascades through a combination of NF-κB activation, increasing reactive oxygen species, and promoting leukocyte recruitment as an adhesion receptor [24]. Enhanced expression of RAGE has been demonstrated in various chronic inflammatory diseases such as diabetes, atherosclerosis, rheumatoid arthritis, and inflammatory kidney disease [25]. Recently, a study by Ihara et al. demonstrated that in diabetic Apo E knockout mice, there was an increased expression of RAGE that was significantly suppressed in diabetic Apo E knockout/Angiotensin II type 1 receptor knockout mice [26]. Since RAGE expression is downregulated after knockout of the angiotensin II type 1 receptor, it is conceivable that angiotensin II activation will result in increased RAGE expression and activity.

This is the first study, to our knowledge, to demonstrate that inhibition of RAGE activation by administration of the RAGE decoy receptor, sRAGE, results in a significant, dose-dependent decrease in angiotensin II induced atherosclerosis formation and improvement in 60 day survival. In this experiment, we used a recombinant sRAGE-Fc fusion protein cloned from a mammalian cell system. As previous studies have shown that soluble protein-Fc fusion proteins dramatic increase in half-life of soluble protein [27] we were able to demonstrate attenuation of atherosclerosis using a much lower dose than previously described [28]. In another published experiment, we have demonstrated the efficacy of 2 µg of the same sRAGE-Fc fusion protein in attenuating lupus nephritis in NZB-WF1 lupus nephritis mice model [29].

The novelty of this finding is the fact that angiotensin II infusion was associated with markedly increased expression of RAGE in the aortas of non-diabetic Apo E knockout mice. RAGE activation is commonly associated with diabetes, a condition that is connected with increased oxidative stress and inflammation. The dose-dependent effects of sRAGE on inhibiting atherosclerosis indicate that RAGE might be important in mediating angiotensin II-induced progression of atherosclerosis. However, the mechanism linking angiotensin II activation with RAGE activation is not defined. We speculate that the increased oxidative stress and inflammation associated with angiotensin II activation results in leukocyte infiltration and cellular necrosis, which will result in increased extracellular release of S100/calgranulin and HMGB1. We showed that RAGE activation acts to increase the degree of inflammation and upregulation of RAGE expression. Although there is a report that S100B stimulates proliferation and migration in vascular smooth muscle through RAGE-mDia1 interaction [30], a mechanism to link angiotensin II activation with RAGE expression is unclear at the present time. The results from our immunohistochemical staining, western blot and RT-PCR analyses demonstrated increased expression of RAGE, ICAM-1, and MCP-1 in the aortas of angiotensin II-administered Apo E knockout mice, all of which were significantly attenuated with sRAGE administration. We also checked systolic and diastolic blood pressure to demonstrate whether or not the effect of sRAGE in AngII is related to regulation of blood pressure as blood pressure could be a factor that could accelerate atherosclerosis independent from the effect of angiotensin II [31]. Although AngII significantly increased blood pressure compared to control, the administration of sRAGE failed to decrease blood pressure when compared to the AngII-infused mouse, suggesting that effects of sRAGE for AngII is independent from blood pressure regulation (Figure 7). Further, it is interesting to note the decreased expression of RAGE was observed in the aortas of animals treated with sRAGE. RAGE is a unique receptor in that it is positively upregulated following ligand activation. As such, the inhibition of RAGE activation by sRAGE may act to attenuate the expression of RAGE as well as the expression of various chemokine and adhesion molecules that are mediated by RAGE activation.

**Figure 7:** Measurement of Mice Blood Pressure. A. The results from the mice tail systolic and B, diastolic blood pressure. Compared to group 1 and group 2 were associated with significant increase in the blood pressure but, between group 2 and group 3 was not significant. N = 7 for each groups. *p<0.05, ns = non-significant.

One of the limitations of this study was the fact that as sRAGE is an indirect inhibitor of RAGE activation acting through binding of RAGE ligands, we cannot rule out the possibility that inhibition of Toll-Like Receptor activation may have contributed to the results. As TLR 2/4 activation can be mediated by RAGE ligands such as HMGB1 [32], sRAGE is not a specific blocker of RAGE activation as the administration of sRAGE may partially inhibit TLR4 activation. This has been demonstrated in a previous experiment demonstrating the efficacy of sRAGE in attenuating atherosclerosis in RAGE KO mice [32]. However, we still believe that sRAGE has a significant effect in blocking RAGE activation because firstly, Liliensiek’s results are limited to adaptive immune responses such as EAE or DTH models [33] and secondly, increased expression of RAGE and inflammatory markers by AngII were significantly reduced under sRAGE treatment in our experiment (Fig. 1C). Further studies using RAGE blocking antibodies or RAGE/Apo E double knockout mouse models will be needed.

In conclusion, the results from this study suggest that RAGE activation may be important in mediating AngII-induced atherosclerosis which was shown to be independent from blood pressure elevation. In addition, as AngII activation is a major pathway in the development of atherosclerosis, the results from this study may provide the basis for future anti-atherosclerotic drug development focused on targeted RAGE activation.
